The article "The Effect of Tibial Insertion Site in Single-Bundle ACL Reconstruction during Gait Based on Motion Capture and Musculoskeletal Model" was published in 2022. Journal: J Healthc Eng.

# The Effect of Tibial Insertion Site in Single-Bundle ACL Reconstruction during Gait Based on Motion Capture and Musculoskeletal Model

**DOI:** 10.1155/2022/7596995

**Published:** 2022-02-26

**Authors:** Xiaotong Li, Yuqing Cao, Xiang Wu, Andrew Merryweather, Haotian Pang, Pengfei Zheng, Hang Xu

**Affiliations:** ^1^School of Medical Imaging, Xuzhou Medical University, Xuzhou, Jiangsu, China; ^2^Department of Mechanical Engineering, University of Utah, Salt Lake, UT, USA; ^3^Department of Orthopaedic Surgery, Children's Hospital of Nanjing Medical University, Nanjing, Jiangsu, China

## Abstract

The purpose of this study was to investigate the effect of tibial insertion site (TIS) of the anterior cruciate ligament (ACL) in single-bundle ACL reconstruction on ligament force during gait. A musculoskeletal model with an ACL ligament was created, and gait data were collected based on the motion capture system from seven female patients with single-bundle ACL reconstruction. The TIS was simulated in OpenSim and systematically changed in 2.5 mm intervals (2.5 mm, 5.0 mm, and 7.5 mm) in the anteroposterior and mediolateral directions from the center. The changes of the ACL force overtime and peak force were compared using the Pearson correlation and paired *t*-test separately for all simulated TISs. The results indicated that anterior movement of the TIS would significantly increase the loading of reconstructed ACL and the risk of secondary injury, but the posterior TIS would keep the ACL loose during gait. The mediolateral change of the TIS also affected the ligament force during gait, which increased in the medial direction and decreased in lateral direction, but the magnitude of the change is relatively small compared with those measured in the anteroposterior direction. Therefore, during preoperative surgery planning, defining the outline of the ACL attachment site during surgery can help to guide the decision for the TIS and can significantly affect the reconstructed ACL force during gait, especially if the TIS is moved in the anteroposterior direction.

## 1. Introduction

The anterior cruciate ligament (ACL) is a key structure in the knee joint, as it resists anterior tibial translation and rotational loads, which are important to maintaining the normal motion and stability of the knee joint. When the distance between the origin of the ACL on the femur and its insertion on the tibia exceeds the threshold of ACL length, ACL tears or injuries could happen, which can significantly affect knee function with subsequent damage to articular cartilage, meniscus, and ultimately lead to joint degeneration and osteoarthritis [1]. The primary treatment for ACL rupture is surgical reconstruction. The annual incidence of ACL tears is 68.6 per 100,000 persons in the United States and 50% of them require ACL reconstruction [2]. Although there are no detailed numbers of ACL ruptures reported in China, the number of patients with ACL reconstruction is increasing every year.

Both single-bundle and double-bundle reconstructions techniques are widely used in the ACL reconstruction surgery. Single-bundle reconstruction is a traditional method, and its ability to restore normal knee function, especially flexion/extension, has been confirmed in multiple studies [3, 4], but whether single-bundle reconstruction can recover the stability of knee rotation is still controversial [5, 6]. Double-bundle reconstruction is a relatively new method which has not only some theoretical advantages but also has challenges due to positioning of the bone tunnel and has a higher risk of femoral epicondyle and bridge fracture compared with single-bundle reconstruction [7]. Additionally, double-bundle reconstruction is not suitable for patients with intercondylar fossa stenosis and the tibial plateau with small anteroposterior diameter [8]. Some previous studies support that double-bundle reconstruction can better recover knee rotation stability than single-bundle reconstruction [9, 10], but others report no significant differences of clinical and functional outcome, the incidence of knee osteoarthritis, and risk of graft failure between these two methods [11–13].

During the process of ACL reconstruction, the damaged ACL is removed and the graft is then replaced; surgeon needs to drill tunnels into the thighbone and shinbone to position and secure the graft. The tunnel location is one of the key factors that influence the force in the reconstructed ACL. It is commonly suggested to place the tunnel in the center of the native femoral insertion site and tibial insertion site (TIS) [4]. However, the consensus on the exact location of the femoral and tibial footprint centers is lacking [14]. Heming et al. described the TIS of the ACL as an 18.5 × 10 mm ellipse and the surgeon should strive toward locating the tunnel approximately at the center of this ellipse [15]. But a certain deviation usually exists between the tunnel location and native tibial footprint of the ACL. The effect of the position achieved during surgery on the ACL function is unclear, and the relationship between the amount of deviation and position from center on ligament force during gait is also largely unknown.

Some previous studies focus on the effect of different femoral insertion sites and TISs for ACL reconstruction mainly based on cadaver specimens [16–18]. Rayan et al. demonstrated that anteroposterior movement of the ACL graft placement within the native femoral footprint of the ACL significantly affects the tension and load distribution on the graft [16]. Markolf et al. reported that the positioning of the femoral tunnel in the anteroposterior direction is more critical than the stress and function of the graft [17]. Edwards et al. investigated the influence of the ACL graft insertion site on the fiber length and reported that moving the TIS in the anteroposterior direction had a significant impact on the length of graft fiber compared with moving in the mediolateral direction during knee flexion [18]. However, it is unclear how changes of the ACL graft at the TIS affect the reconstructed ligament force during functional movements. Therefore, the purpose of this study was to investigate the influence of the TIS in single-bundle ACL reconstruction on ligament force during gait. We hypothesized that the TIS in the anteroposterior direction would largely affect the ACL force during gait, but would not significantly alter the force if located medial or lateral from the center position. The implications of this work could influence how surgeons decide where to place the TIS during single-bundle ACL reconstruction.

## 2. Methodology

### 2.1. Musculoskeletal Model

The musculoskeletal model developed in this study was based on a previous OpenSim model (available at https://simtk.org/projects/kneeligament) [19]; our model consisted of 12 rigid segments, 92 muscle actuators, and 27 DOFs (degrees of freedom), including 3 DOFs for trunk, 6 DOFs for pelvis, 3 DOFs for hip joints, 3 DOFs for knee joints, and 1 DOF for ankle, subtalar, and metatarsophalangeal joint, respectively. The femur reference frame was fixed at the center of the femoral head, and the tibial reference frame was located at the midpoint of the line between the medial and lateral femoral epicondyles. For both femur and tibial reference coordination, the *x*-axis pointed anteriorly, the *y*-axis pointed proximally, and the *z*-axis pointed laterally. The knee rotations in three body planes were all independent, but the anteroposterior transformations between femur and tibia were defined as a function of knee flexion.

### 2.2. Definition of ACL Parameters

An elastic element was used to describe the geometric and mechanical behaviour of the ACL in our model. The path of the ACL is considered as a straight line, as shown in Figure 1. The initial values of ACL parameters, such as the femoral insertion site and TIS, stiffness, and resting length (Table 1) were obtained from literature [20], as given in Table 1.

The tension of the ACL was a function of its length, and the force-strain curve was defined by a nonlinear step-wise function for low strains and a linear function for strains higher than a certain level as [20]

(1) $$\begin{array}{c} f_{l}=\left\{\begin{array}{cc} 0, & e\leq 0,\\ \frac{0.25*k*e^{2}}{e_{l}}, & 0\leq e\leq 2e_{l},\\ k\left(e-e_{l}\right), & e\geq 2e_{l}, \end{array}\right. \end{array}$$

where *k* is the ligament stiffness, *e*_*l*_ is the linear strain limit which was set at 0.03, and *e* is the ligament strain which is calculated by

(2) $$\begin{array}{c} e=\frac{L-L_{0}}{L_{0}}, \end{array}$$

where *L* is the ligament length and *L*_0_ is the resting length of ligament.

### 2.3. Gait Data Collection

Seven female patients with unilateral single-bundle ACL reconstruction and no other history of serious lower limb injury were recruited from a local hospital (30.86 ± 11.79 years old, height of 1.63 ± 0.98 m, body mass of 72.04 ± 15.22 kg, and BMI of 27.12 ± 4.42 kg/m^2^). All participants had a single-bundle ACL reconstruction performed with a standard transtibial technique using a patellar tendon allograft. The gait data were collected after 6 months postreconstruction in the Biomechanics and Motion Analysis Laboratory at Xuzhou Medical University. 14 mm reflective markers were attached to the participants based on the Conventional Gait Model 2.3 marker set [21]. The marker trajectories and ground reaction forces were recorded using a ten-camera motion capture system at 100 Hz (Vicon Motion Systems Ltd., Oxford, UK) and two force plates at 1000 Hz (Advanced Mechanical Technology Inc., Watertown, USA), respectively. Institutional review board approval was obtained, and all participants reviewed and signed an informed consent document.

### 2.4. Gait Simulation and Estimation of ACL Force

OpenSim is an open-source platform for modelling, simulating, and analyzing the musculoskeletal system. OpenSim 4.0 software was used to simulate the gait and estimate the ACL force. The musculoskeletal model was first scaled to each participant based on a comparison of experimental marker data with virtual markers placed on the model using the static trial. The ligament geometry and resting length of the ACL were also scaled except for the stiffness. Then, joint kinematics in each time step were determined by a weighted least squares approach to best match the experimental markers during gait. Finally, the static optimization algorithm was recruited to solve the net joint moments into the muscle and ACL forces to drive the dynamic gait simulation [22].

### 2.5. Evaluation of ACL Force by Different TISs

In order to evaluate the ACL force at different TISs for a single-bundle ACL reconstruction, the femoral insertion site in the model was kept constant for each participant after scaling, but the TIS was systematically changed in 2.5 mm intervals (2.5 mm, 5.0 mm, and 7.5 mm) in medial/lateral and anterior/posterior directions based on the initial cantered ellipse for the TIS located, as shown in Figure 2. Gait data from each participant were simulated 13 times for each participant to obtain the ACL forces for different TISs. Gait data were normalized to 101 points for each gait cycle.

### 2.6. Statistical Analysis

The statistical analyses were performed using SPSS 20 (IBM Corporation, Armonk, NY). The correlation of ACL force curves between center position and other TISs were determined using Pearson correlation. The magnitudes of the peak ACL force in the stance phase were compared between center position and the other 12 TISs in four directions separately using the paired *t*-test. The results were considered statistically significant when *P* < 0.05.

## 3. Results

### 3.1. Knee Kinematics

The average knee kinematics for the ACL reconstruction limb during gait are shown in Figure 3. The maximum knee flexion angles were 14 degrees and 64 degrees in the stance and swing phases, respectively. The peak of knee adduction angle was 10 degrees around 85% of the gait cycle, and the maximum knee internal and external rotations in the swing phase were 7 degrees and 12 degrees, respectively.

### 3.2. The Change of ACL Force Curve by Different TISs

The ACL force curves changed with different TISs and are shown in Figure 4. The correlation analyses indicated that ACL force curves still had high correlation (*P* < 0.01) when the TIS changed 2.5 mm from center except for three subjects in the posterior direction, as given in Table 2. The correlation decreased followed by the increased distance when the TIS moved anteriorly, medially, and laterally from center. There were no ACL forces generated during gait when the TIS was located posteriorly 5.0 mm or 7.5 mm from the center.

Two peaks of the ACL force were observed in the stand phase which happened at the initial contact and terminal stance separately. The peak ACL forces increased when the TIS moved anteriorly and medially, but decreased when the TIS moved laterally, as given in Table 3. Significant differences were observed in the corresponded peak ACL forces between center position and the changed TIS (*P* < 0.05).

## 4. Discussion

The ACL forces during gait after ACL reconstruction were largely dependent on the knee kinematics. After six months recovery, the knee motions in three body planes for the ACL reconstruction patients in our study were similar to the normal knee kinematics curves during gait reported by previous research [23].

Cadaver studies report that the ultimate force of the ACL varied between 600 and 2300 N based on experiments of the ACL with bone supports, such as the femur-ACL-tibia complex [24]. The change in the TIS within 7.5 mm from the center position still produced the peak ACL force during gait (551 N for 7.5 mm in anterior direction, Table 3) below the ultimate force. However, the ACL strain in functional activities is usually between 1/4 and 1/3 of ultimate strain [25], and the anterior movement of the TIS (such as 5.0 mm and 7.5 mm) would increase the required load of the reconstructed ACL and also the risk of secondary injury. A surgeon should be aware of the effects of the TIS position during ACL reconstruction, especially in the anterior direction, due to the significant increase in the ACL force compared to the center position (Figure 4). We also observed that the function of the ACL quickly disappeared and even remained in a slack state during the whole gait cycle when the TIS moved posteriorly above 2.5 mm. This finding aligned with previous conclusion that the TIS for ACL reconstruction should not be around the posterior limit of the original ACL, which could avoid vertical graft placement and better match the function of the ACL [26, 27].

During the gait cycle, the ACL force increased when the TIS moved medially and decreased when the TIS moved laterally (Figure 4). The correlations were relatively high when the TIS changed medially from center (Table 2). Previous computational studies reported the pattern of loading on the ACL during the gait cycle and showed the peak ACL force between 156 and 411 N at early stance [28], which was larger than the peak ACL force when the TIS was in the center (71.47 N in Table 3). This finding implied that the center position of the TIS may be not always the best choice during surgery. Moving the TIS medially rather than anteriorly may be a better option, since the magnitude of the change is less sensitive in the medial direction than in the anteroposterior direction.

High-resolution MRI analysis confirm that the original ACL TIS is elliptical or triangular in healthy knees and the size of the TIS varies greatly [26, 29], which require a surgeon to outline the size and shape of the ACL attachment in each patient making it challenging to standardize the optimal position of the TIS in ACL reconstruction. The shape of the ACL TIS is determined based on the width of the midsubstance with the help of high-resolution MRI analysis. The hypothesis that the TIS in anteroposterior direction could largely affect the ACL force during gait but not in the mediolateral direction was supported in the present study. Our results were similar to the findings for the femur insertion site in ACL reconstruction, which implied that placement of a graft too far in an anterior or a posterior position had a large effect on deleterious lengthening and graft failure [16, 17].

Some limitations existed in the present study. First, the original insertion sites of the ACL in the femur and tibia in the present musculoskeletal model were derived from specimen studies. Therefore, the insertion site differences between participants and the model might exist. However, the function of the ACL in the musculoskeletal model has been validated in a previous research [19]. Therefore, it should not affect the tendency of the ACL force changes when the TIS deviated from center. Second, the resting length was constant in the musculoskeletal model and derived from the literature in our study. But it could be different for each participant. Although the resting length could be determined by the reference strain and reference length, the reference strain was not measured in vivo.

## 5. Conclusion

This study demonstrated that the position of the TIS in single-bundle ACL reconstruction can significantly affect the ACL force generated during gait. The results suggest that anterior movement of the TIS from a center position would increase the ACL force significantly, but posterior deviation of the TIS would keep the ACL loose and inhibit function during gait. Mediolateral movement of the TIS can also affect the ACL force during gait, which was increased in the medial direction and decreased in lateral direction, but the magnitude of change is relatively mild compared with the anteroposterior direction. Therefore, surgeons should outline the size and shape of the ACL attachment region in single-bundle ACL reconstruction and center the TIS as closely as possible to the anatomic attachment point, especially in the anteroposterior direction. Future work should consider defining a method for surgeons to more easily define these anatomical regions to improve surgical outcomes.

## Figures and Tables

**Figure 1:** The location and attachments of the ACL in the musculoskeletal model.

**Figure 2:** The placement of the TIS of a reconstructed ACL. The blue oval represents the anatomical area of the TIS for the ACL, the small black dot represents the center position, and the small red dots represent the different TISs.

**Figure 3:** The average knee kinematics for the ACL reconstruction limb during gait. The shaded regions indicated the standard deviation of knee kinematics.

**Figure 4:** The average ACL force curves for 2.5 mm, 5.0 mm, and 7.5 mm TISs from the center. The shaded regions indicated standard deviation of the ACL force when the TIS was in the center.

**Table 1:** The initial ACL parameters in the musculoskeletal model.

	Femoral insertion site (cm)			Tibial insertion site (cm)			Resting length (cm)	Stiffness (N)
	*X*	*Y*	*Z*	*X*	*Y*	*Z*		
ACL	−1.1	−40.5	0.7	1.2	−3.2	−0.1	2.8	3100

**Table 2:** Correlation of the ACL force curve between center and changed TIS.

	Anterior			Posterior		
	2.5 mm	5.0 mm	7.5 mm	2.5 mm	5.0 mm	7.5 mm
Subject 01	0.935^*∗∗*^	0.851^*∗∗*^	0.850^*∗∗*^	0.870^*∗∗*^	N/A	N/A
Subject 02	0.942^*∗∗*^	0.882^*∗∗*^	0.878^*∗∗*^	0.859^*∗∗*^	N/A	N/A
Subject 03	0.800^*∗∗*^	0.504^*∗*^	0.470^*∗*^	0.797^*∗∗*^	N/A	N/A
Subject 04	0.863^*∗∗*^	0.753^*∗∗*^	0.747^*∗∗*^	0.594^*∗*^	N/A	N/A
Subject 05	0.837^*∗∗*^	0.681^*∗*^	0.664^*∗*^	0.573^*∗*^	N/A	N/A
Subject 06	0.870^*∗∗*^	0.791^*∗∗*^	0.809^*∗∗*^	0.712^*∗∗*^	N/A	N/A
Subject 07	0.879^*∗∗*^	0.792^*∗∗*^	0.660^*∗*^	0.670^*∗*^	N/A	N/A
Mean	0.875	0.75	0.726	0.725	N/A	N/A

	Medial			Lateral		
	2.5 mm	5.0 mm	7.5 mm	2.5 mm	5.0 mm	7.5 mm
Subject 01	0.973^*∗∗*^	0.881^*∗∗*^	0.837^*∗∗*^	0.961^*∗∗*^	0.925^*∗∗*^	0.828^*∗∗*^
Subject 02	0.976^*∗∗*^	0.932^*∗∗*^	0.905^*∗∗*^	0.957^*∗∗*^	0.842^*∗∗*^	0.616^*∗*^
Subject 03	0.942^*∗∗*^	0.703^*∗∗*^	0.600^*∗*^	0.956^*∗∗*^	0.933^*∗∗*^	0.796^*∗∗*^
Subject 04	0.880^*∗∗*^	0.730^*∗∗*^	0.594^*∗*^	0.869^*∗∗*^	0.745^*∗∗*^	0.658^*∗*^
Subject 05	0.901^*∗∗*^	0.723^*∗∗*^	0.650^*∗*^	0.893^*∗∗*^	0.851^*∗∗*^	0.631^*∗*^
Subject 06	0.938^*∗∗*^	0.814^*∗∗*^	0.706^*∗∗*^	0.956^*∗∗*^	0.906^*∗∗*^	0.852^*∗∗*^
Subject 07	0.956^*∗∗*^	0.849^*∗∗*^	0.551^*∗*^	0.965^*∗∗*^	0.909^*∗∗*^	0.879^*∗∗*^
Mean	0.938	0.805	0.692	0.937	0.873	0.751

^*∗∗*^Significant correlation at 0.01 level. ^*∗*^Significant correlation at 0.05 level. N/A, no ACL force generated at these positions during gait.

**Table 3:** The peak ACL forces in the stance phase.

Center		First peak (N)	Second peak (N)
		71.47 ± 26.78	59.81 ± 23.27
2.5 mm	Anterior	207.83 ± 25.89	196.88 ± 28.74^*∗*^
	Posterior	8.11 ± 2.13^*∗*^	3.87 ± 1.28^*∗*^
	Medial	139.76 ± 25.40^*∗*^	126.16 ± 27.54^*∗*^
	Lateral	30.95 ± 12.25^*∗*^	27.79 ± 9.11^*∗*^

5.0 mm	Anterior	383.82 ± 28.64^*∗*^	376.31 ± 29.72^*∗*^
	Posterior	N/A	N/A
	Medial	253.2 ± 28.53^*∗*^	233.14 ± 32.55^*∗*^
	Lateral	19.04 ± 7.11^*∗*^	17.03 ± 6.92^*∗*^

7.5 mm	Anterior	551.36 ± 34.43^*∗*^	546.83 ± 36.90^*∗*^
	Posterior	N/A	N/A
	Medial	325.55 ± 38.02^*∗*^	339.56 ± 38.65^*∗*^
	Lateral	10.43 ± 4.79^*∗*^	10.55 ± 4.38^*∗*^

^*∗*^Significant difference of peak ACL force compared with center position, *P* < 0.05.

## Data Availability

The datasets used and/or analyzed during the current study are available from the corresponding author upon request.
